RETRACTED

# Open Nephroureterectomy Compared to Laparoscopic in Upper Urinary Tract Urothelial Carcinoma: A Meta-Analysis

**DOI:** 10.3389/fsurg.2021.729686

**Published:** 2021-08-13

**Authors:** Guihong Liu, Zeqin Yao, Guoqiang Chen, Yalang Li, Bing Liang

**Affiliations:** ^1^Department of Urology, Sanya Central Hospital (Hainan Third People's Hospital), Sanya, China; ^2^Department of Urology, Yuzhou People's Hospital, Xuchang, China

**Keywords:** open nephroureterectomy, laparoscopic, upper urinary tract urothelial carcinoma, complications, perioperative results, survival

## Abstract

**Background:** In this meta-analysis, we will focus on evaluating the effects of open nephroureterectomy compared with laparoscopic nephroureterectomy on postoperative results in upper urinary tract urothelial carcinoma subjects.

**Methods:** A systematic literature search up to January 2021 was performed, and 36 studies included 23,013 subjects with upper urinary tract urothelial carcinoma at the start of the study; of them, 8,178 were laparoscopic nephroureterectomy, and 14,835 of them were open nephroureterectomy. They were reporting relationships between the efficacy and safety of open nephroureterectomy compared with laparoscopic nephroureterectomy in the treatment of upper urinary tract urothelial carcinoma. We calculated the odds ratio (OR) or the mean difference (MD) with 95% CIs to evaluate the efficacy and safety of open nephroureterectomy compared with laparoscopic nephroureterectomy in the treatment of upper urinary tract urothelial carcinoma using the dichotomous or continuous method with a random or fixed-effect model.

**Results:** Laparoscopic nephroureterectomy in subjects with upper urinary tract urothelial carcinoma was significantly related to longer operation time (MD, 43.90; 95% CI, 20.91–66.90, *p* < 0.001), shorter hospital stay (MD, −1.71; 95% CI, −2.42 to −1.00, *p* < 0.001), lower blood loss (MD, −133.82; 95% CI, −220.92 to −46.73, *p* = 0.003), lower transfusion need (OR, 0.56; 95% CI, 0.47–0.67, *p* < 0.001), and lower overall complication (OR, 0.79; 95% CI, 0.70–0.90, *p* < 0.001) compared with open nephroureterectomy.

However, no significant difference was found between laparoscopic nephroureterectomy and open nephroureterectomy in subjects with upper urinary tract urothelial carcinoma in 2–5 years recurrence-free survival (OR, 0.90; 95% CI, 0.69–1.18, *p* = 0.46), 2–5 years cancer-specific survival (OR, 0.94; 95% CI, 0.69–1.28, *p* = 0.68), and 2–5 years overall survival (OR, 1.31; 95% CI, 0.91–1.87, *p* = 0.15).

**Conclusion:** Laparoscopic nephroureterectomy in subjects with upper urinary tract urothelial carcinoma may have a longer operation time, shorter hospital stay, and lower blood loss, transfusion need, and overall complication compared to open nephroureterectomy. Further studies are required to validate these findings.

RETRACTED

## Background

Urothelial carcinoma of the upper urinary tract is a rare type of malignancy with 1–5% of all urological cancers (1). Because synchronous or metachronous tumors are an inherited behavior of urothelial cancer, radical nephroureterectomy, the bladder cuff excision is considered the standard management for urothelial carcinoma of the upper urinary tract, particularly for muscle-invasive and/or high-grade carcinoma (2). Of present, open nephroureterectomy is the most frequently used procedure for urothelial carcinoma of the upper urinary tract with high risk. Though open nephroureterectomy has been shown to produce long-term local control and improve survival, it may be related to significant morbidity (2). Meanwhile, the first laparoscopic nephroureterectomy was executed in 1993 (3). Minimally invasive methods have rapidly advanced, and laparoscopic surgery of the upper urinary tract has turned into an accepted method by urological surgeons (4). Laparoscopic nephroureterectomy is similarly in effect as open nephroureterectomy surgery for urothelial carcinoma of the upper urinary tract, though causing less perioperative morbidity; as urothelial carcinoma of the upper urinary tract is an aggressive malignancy with a high possibility for disease reappearance and mortality. It is hypothesized that cancer cell dissemination and high-pressure pneumoperitoneum throughout laparoscopic nephroureterectomy could be related to a higher risk of bladder cancer, local recurrence, and port-site metastasis (5). So, the oncologic efficiency of laparoscopic nephroureterectomy compared with open nephroureterectomy remains conflicting. Several studies have compared the results of laparoscopic nephroureterectomy and open nephroureterectomy for urothelial carcinoma of the upper urinary tract. Yet, the role of laparoscopic nephroureterectomy is not recognized (6). The surgical practice and experience have developed much since the first laparoscopic nephroureterectomy procedure (3). So, we performed this meta-analysis study to assess the efficacy and safety of open nephroureterectomy compared with laparoscopic nephroureterectomy in the treatment of upper urinary tract urothelial carcinoma.

## Methods

The present study followed the meta-analysis of studies in the epidemiology statement (7), which was performed following an established protocol.

### Study Selection

Studies included were those with statistical measures of association [odds ratio (OR), mean difference (MD), frequency rate ratio, or relative risk, with 95% CIs) between the efficacy and safety of open nephroureterectomy compared with laparoscopic nephroureterectomy in the treatment of upper urinary tract urothelial carcinoma.

RETRACTED

Human studies only in the English language were considered. Inclusion was not restricted by size or type of study. Publications excluded were review articles and commentary and studies that did not supply a degree of relationship. Figure 1 shows the whole study process.

**Figure 1:** Schematic diagram of the study procedure.

The articles were integrated into the meta-analysis when the following inclusion criteria were met:

1. The study was a randomized controlled trial or retrospective study.

2. The target population is subjects with upper urinary tract urothelial carcinoma.

3. The intervention program was the open nephroureterectomy and laparoscopic nephroureterectomy.

4. The study included comparisons between the efficacy and safety of open nephroureterectomy compared with laparoscopic nephroureterectomy in the treatment of upper urinary tract urothelial carcinoma.

The exclusion criteria were the following:

1. Studies that did not compare open nephroureterectomy to laparoscopic nephroureterectomy.

2. Studies with surgery other than upper urinary tract urothelial carcinoma.

3. Studies did not concentrate on the effect on postoperative results.

### Identification

A search protocol strategy was organized according to the PICOS principle (8), and we defined it as follow: P (population): subjects with upper urinary tract urothelial carcinoma; I (intervention/exposure): open nephroureterectomy and laparoscopic nephroureterectomy; C (comparison): efficacy and safety of open nephroureterectomy compared with laparoscopic nephroureterectomy in the treatment of upper urinary tract urothelial carcinoma; O (outcome): perioperative, and postoperative results; S (study design): no restriction (9). First, we conducted a systematic search of Embase, PubMed, Cochrane Library, OVID, and Google scholar till January 2021, by a blend of keywords and related words for open nephroureterectomy, laparoscopic, upper urinary tract urothelial carcinoma, complications, perioperative results, and survival as shown in Table 1. All selected studies were gathered in an EndNote file, duplicates were removed, and the title and abstracts were revised to eliminate studies that did not report the relationship between the efficacy and safety of open nephroureterectomy compared with laparoscopic nephroureterectomy in the treatment of upper urinary tract urothelial carcinoma. The remaining studies were examined for related information.

**Table 1:** Search strategy for each database.

**Database**	**Search strategy**
Pubmed	#1 “open nephroureterectomy”[MeSH Terms] OR “laparoscopic”[All Fields] OR “upper urinary tract urothelial carcinoma”[All Fields] #2 “complications”[MeSH Terms] OR “open nephroureterectomy”[All Fields] OR “postoperative results”[All Fields] OR “survival”[All Fields] #3 #1 AND #2
Embase	'open nephroureterectomy'/exp OR 'laparoscopic'/exp OR 'upper urinary tract urothelial carcinoma'/exp #2 'complications'/exp OR 'ICBG'/exp OR 'postoperative results' OR 'survival' #3 #1 AND #2
Cochrane library	#1 (open nephroureterectomy):ti,ab,kw OR (laparoscopic):ti,ab,kw OR (upper urinary tract urothelial carcinoma):ti,ab,kw (Word variations have been searched) #2 (complications):ti,ab,kw OR (postoperative results):ti,ab,kw OR (survival):ti,ab,kw (Word variations have been searched) #3 #1 AND #2

RETRACTED

### Screening

Data were abbreviated based on the following: study associated and subject associated features onto a homogeneous form. We extracted the following data separately: the last name of the primary author, study period, publication year, country, the studies region, and design of the study; type of the population, the total number and subjects number, demographic data, and clinical and treatment features; the evaluation period associated with measurement, quantitative method and qualitative method of assessment, source of information, and assessment of outcomes; and statistical analysis MD or relative risk, with 95% CI of the relationship between efficacy and safety of open nephroureterectomy compared with laparoscopic nephroureterectomy in the treatment of upper urinary tract urothelial carcinoma (10). If a study fit for inclusion based upon the above-mentioned principles, data were extracted individually by two authors. In case of discrepancy, the corresponding author gave a final choice. When there were diverse data from a study, the data were extracted separately. In case of bias risk in the studies, each study was assessed using two authors who individually evaluated the methodological quality of the selected studies. We used the “risk of bias tool” from the RoB 2: a revised Cochrane risk-of-bias tool for randomized trials to evaluate methodological quality (11). In terms of the evaluation criteria, each study was valued and allocated to one of the next three risks of bias: low: if all quality criteria were met; unclear or moderate: if one or more of the quality criteria were partly met or unclear; high: if one or more of the criteria were not met, or not included. Any discrepancies were addressed by a reassessment of the original article.

### Eligibility

The main result concentrated on the efficacy and safety of open nephroureterectomy compared with laparoscopic nephroureterectomy in the treatment of upper urinary tract urothelial carcinoma. An assessment of the efficacy and safety of open nephroureterectomy compared with laparoscopic nephroureterectomy in the treatment of upper urinary tract urothelial carcinoma was extracted forming a summary.

RETRACTED

### Inclusion

Sensitivity analyses were limited only to studies reporting the relationship between the efficacy and safety of open nephroureterectomy compared with laparoscopic nephroureterectomy in the treatment of upper urinary tract urothelial carcinoma. For subcategory and sensitivity analysis, we compared the effect of open nephroureterectomy compared with laparoscopic nephroureterectomy.

### Statistical Analysis

The dichotomous or continuous method with random-effect or fixed-effect models was used to calculate the OR or MD and 95% CI. We used the Chi-squared test to perform biological heterogeneity analyses between different studies. We calculated the *I*^2^ index, and the *I*^2^ index is from 0 to 100%. Values of about 0%, 25%, 50%, and 75% indicate no, low, moderate, and high heterogeneity, respectively (8). When *I*^2^ was higher than 50%, we chose the random effect model; when it was lower than 50%, we used the fixed-effect model. A subgroup analysis was performed by stratifying the original evaluation per liver cancer and different outcomes of chemotherapy as described before. In this analysis, a *p*-value for differences between subgroups of <0.05 was considered statistically significant. Publication bias was evaluated quantitatively using the Egger regression test (publication bias considered present if *p* ≥ 0.05), and qualitatively, by visual examination of funnel plots of the logarithm of ORs or MDs vs. their SE (10). All *p*-values were two-tailed. All calculations and graphs were performed using Reviewer manager version 5.3 (The Nordic Cochrane Center, The Cochrane Collaboration, Copenhagen, Denmark).

## Results

A total of 2,534 unique studies were identified, of which 36 studies (between 2007 and 2020) fulfilled the inclusion criteria and were included in the study (12–47).

The 36 studies included 23,013 subjects with upper urinary tract urothelial carcinoma at the start of the study, 8,178 of them were laparoscopic nephroureterectomy, and 14,835 of them were open nephroureterectomy. All studies evaluated the efficacy and safety of open nephroureterectomy compared with laparoscopic nephroureterectomy in the treatment of upper urinary tract urothelial carcinoma.

Study size ranged from 26 to 3,984 subjects with upper urinary tract urothelial carcinoma at the start of the study. The details of the 36 studies are shown in Table 2. About 16 studies reported data stratified to operation time, 13 studies stratified to the hospital stay, 10 studies stratified to the blood loss, 5 studies stratified to transfusion need, 10 studies stratified to the overall complication, 25 studies stratified to the 2–5 years recurrence-free survival, 28 studies reported data stratified to studies stratified to 2–5years cancer-specific survival, and 20 studies reported data stratified to 2–5 years overall survival.

RETRACTED

**Table 2:** Characteristics of the selected studies for the meta-analysis.

**Study**	**Country**	**Total**	**Laparoscopic nephroureterectomy**	**Open nephroureterectomy**
Koda et al. (12)	Japan	106	79	27
Manabe et al. (13)	Japan	224	58	166
Rouprêt et al. (14)	France	46	20	26
Hemal et al. (15)	USA	48	21	27
Taweemonkongsap et al. (16)	Thailand	60	31	29
Terakawa et al. (17)	Japan	240	120	120
Capitanio et al. (18)	Multicenter	1,249	270	979
Greco et al. (19)	Germany	140	70	70
Simone et al. (20)	Italy	80	40	40
Waldert et al. (21)	Austria	102	43	59
Favaretto et al. (22)	USA	162	53	109
Stewart et al. (23)	UK	62	23	39
Walton et al. (24)	Multicenter	773	70	703
Ariane et al. (25)	France	609	150	459
Metcalfe et al. (26)	USA	849	446	403
Fairey et al. (27)	Canada	849	446	403
Xylinas et al. (28)	France	482	132	350
Fradet et al. (29)	Canada	612	345	267
Kitamura et al. (30)	Japan	99	65	34
Zou et al. (31)	China	122	21	101
Blackmur et al. (32)	UK	26	13	13
Hanske et al. (33)	Germany	896	599	297
Kim et al. (34)	Korea	372	100	272
Miyazaki et al. (35)	Japan	849	222	627
Liu et al. (36)	China	265	52	213
Abe et al. (37)	Japan	214	114	100
Kido et al. (38)	Japan	426	75	351
Kim et al. (39)	Korea	1,521	615	906
Lee et al. (40)	Korea	298	137	161
Kim et al. (41)	Korea	1,693	715	978
Nazzani et al. (42)	Multicenter	3,897	1,093	2,804
Shigeta et al. (43)	Japan	176	72	104
Alothman et al. (44)	Saudi Arabia	50	24	26
Ye et al. (45)	China	48	24	24
Azawi et al. (46)	Denmark	1,384	1,063	321
Moschini et al. (47)	Multicenter	3,984	757	3,227
	**Total**	**23,013**	**8,178**	**14,835**

Laparoscopic nephroureterectomy in subjects with upper urinary tract urothelial carcinoma was significantly related to longer operation time (MD, 43.90; 95% CI, 20.91–66.90, *p* < 0.001) with high heterogeneity (*I*^2^ = 98%), shorter hospital stay (MD, −1.71; 95% CI, −2.42 to −1.00, *p* < 0.001) with high heterogeneity (*I*^2^ = 98%), lower blood loss (MD, −133.82; 95% CI, −220.92 to −46.73, *p* = 0.003) with high heterogeneity (*I*^2^ = 96%), lower transfusion need (OR, 0.56; 95% CI, 0.47–0.67, *p* < 0.001) with low heterogeneity (*I*^2^ = 42%), and lower overall complication (OR, 0.79; 95% CI, 0.70–0.90, *p* < 0.001) with low heterogeneity (*I*^2^ = 28%) compared with open nephroureterectomy as shown in Figures 2–6.

RETRACTED

**Figure 2:** Forest plot of the effect of open nephroureterectomy compared with laparoscopic nephroureterectomy on operation time in subjects with upper urinary tract urothelial carcinoma.

**Figure 3:** Forest plot of the effect of open nephroureterectomy compared with laparoscopic nephroureterectomy on hospital stay in subjects with upper urinary tract urothelial carcinoma.

**Figure 4:** Forest plot of the effect of open nephroureterectomy compared with laparoscopic nephroureterectomy on blood loss in subjects with upper urinary tract urothelial carcinoma.

**Figure 5:** Forest plot of the effect of open nephroureterectomy compared with laparoscopic nephroureterectomy on transfusion need in subjects with upper urinary tract urothelial carcinoma.

**Figure 6:** Forest plot of the effect of open nephroureterectomy compared with laparoscopic nephroureterectomy on overall complication in subjects with upper urinary tract urothelial carcinoma.

However, no significant difference was found between laparoscopic nephroureterectomy and open nephroureterectomy in subjects with upper urinary tract urothelial carcinoma in 2–5 years recurrence-free survival (OR, 0.90; 95% CI, 0.69–1.18, *p* = 0.46) with high heterogeneity (*I*^2^ = 89%), 2–5 years cancer-specific survival (OR, 0.94; 95% CI, 0.69–1.28, *p* = 0.68) with high heterogeneity (*I*^2^ = 89%), and 2–5 years overall survival (OR, 1.31; 95% CI, 0.91–1.87, *p* = 0.15) with high heterogeneity (*I*^2^ = 91%) as shown in Figures 7–9.

**Figure 7:** Forest plot of the effect of open nephroureterectomy compared with laparoscopic nephroureterectomy on 2–5 years recurrence-free survival in subjects with upper urinary tract urothelial carcinoma.

**Figure 8:** Forest plot of the effect of open nephroureterectomy compared with laparoscopic nephroureterectomy on 2–5 years cancer-specific survival in subjects with upper urinary tract urothelial carcinoma.

**Figure 9:** Forest plot of the effect of open nephroureterectomy compared with laparoscopic nephroureterectomy on blood loss in subjects with upper urinary tract urothelial carcinoma.

Selected studies stratified analysis that did and did not adjust for age, ethnicity, and the effect of different laparoscopic nephroureterectomy procedures between the two groups was not performed since no studies reported or adjusted for these factors.

Based on the visual examination of the funnel plot as well as on quantitative measurement by the Egger regression test, there was no indication of publication bias (*p* = 0.85). Though, most of the comprised studies were evaluated to be of a low methodological quality. All studies did not have selective reporting bias, and no articles had incomplete result data and selective reporting.

RETRACTED

## Discussion

This meta-analysis study based on 36 studies included 23,013 subjects with upper urinary tract urothelial carcinoma at the start of the study; 8,178 of them were laparoscopic nephroureterectomy, and 14,835 of them were open nephroureterectomy (12–47). Laparoscopic nephroureterectomy in subjects with upper urinary tract urothelial carcinoma may have a longer operation time, shorter hospital stay, and lower blood loss, transfusion need, and overall complication compared with open nephroureterectomy; however, no significant difference was found between laparoscopic nephroureterectomy and open nephroureterectomy in subjects with upper urinary tract urothelial carcinoma in 2–5 years recurrence-free survival, 2–5 years cancer-specific survival, and 2–5 years overall survival (12–47). Though the analysis of outcomes should be done with caution because of the low number of subjects in some of the studies evaluating each parameter in this meta-analysis, suggesting more studies relating the type of operation method, and postoperative results in subjects with upper urinary tract urothelial carcinoma to validate these findings. The need for more studies is very obvious in the results of 2–5 years overall survival with their low *p*-values (*p* = 0.15), showing the need for further research possibly to significantly influence confidence in the effect evaluation.

From the time of the first study comparing open nephroureterectomy with laparoscopic nephroureterectomy in 1993 (3), many studies have tried to show laparoscopic nephroureterectomy as a possible substitute of open nephroureterectomy for urothelial carcinoma of the upper urinary tract, however, there was no comprehensive comparison found. This present meta-analysis with its high-level results establishes a role of laparoscopic nephroureterectomy in the surgical management of urothelial carcinoma of the upper urinary tract. The procedure of laparoscopic nephroureterectomy involves nephrectomy and distal ureterectomy, with the same ontological value as open nephroureterectomy. Laparoscopic access could be done through transperitoneal or retroperitoneal spaces. Transperitoneal access gives more working space and easier handling, while retroperitoneal access avoids disturbance of the intraperitoneal organs and the risk of intraperitoneal corruption by malignant cells (48); however, the process of laparoscopic nephroureterectomy has not been standardized yet, particularly management of the distal ureter. Numerous disposal methods have been designated in the clinical trials, e.g., open surgery (14, 21), the Pluck technique (24, 25), and the LigaSure Atlas system (20). Open surgery is still the most prevalent for bladder cuff excision; however, no significant difference in oncological results was shown between different methods (49).

RETRACTED

As a mini-invasive technique, laparoscopic nephroureterectomy has been accepted over the world as a promising alternative, with some advantages over open nephroureterectomy as shown in this meta-analysis, e.g., less blood loss, less requirement of transfusion, less overall complication, and shorter hospital stay (50–52). This may be due to the large cuts necessary even in laparoscopic nephroureterectomy for the removal of separated samples as well as bladder cuff. Formerly, it was proven that in invasive or large tumors, surgeons should avoid laparoscopic nephroureterectomy (2). With the improvement in methodology and experience of surgeons, the criteria of laparoscopic nephroureterectomy have been intensely expanded. Subjects with high stages (T3/T4) and high grades (G3) experienced laparoscopic nephroureterectomy with similar oncological results as open nephroureterectomy (50–52). Even though different methodology, the oncological values of surgical management of urothelial carcinoma of the upper urinary tract were similar (50–52), and the high risk of regional recurrence and port-site metastasis in laparoscopic nephroureterectomy is still high. Kondo et al. (53) showed that template-based lymphadenectomy decreases the risk of regional lymph node recurrence between subjects with upper/middle ureteral tumor, though templated lymphadenectomy is hard for laparoscopic methodology (54). Xylinas et al. (55) also showed that laparoscopic methodology was an independent risk factor of intravesical recurrence, due to the high pressure that may activate cancer spread (53). Ariane et al. (25) showed a significant number of port-side metastasis with the laparoscopic nephroureterectomy (25); however, other studies showed that surgical methods did not affect postoperative recurrence or survival (55–57). Several meta-analyses have compared laparoscopic nephroureterectomy with open nephroureterectomy, and laparoscopic nephroureterectomy revealed improvement in cancer-specific survival and extravesical recurrence-free survival (6, 50–52); However, either the 5-year survival or the 2-year survival variables did not differ much between laparoscopic nephroureterectomy and open nephroureterectomy.

This meta-analysis reported the relationship between the type of different surgical techniques and postoperative results in subjects with upper urinary tract urothelial carcinoma. Though, additional studies are required to confirm these possible relationships. Similarly, additional studies are required to deliver a clinically meaningful difference in perioperative and postoperative results in subjects with upper urinary tract urothelial carcinoma. These studies must include larger homogeneous samples. This was also recommended in earlier similar meta-analysis studies which showed a similar result of laparoscopic nephroureterectomy and open nephroureterectomy on perioperative and postoperative results in subjects with upper urinary tract urothelial carcinoma (50, 51). Well-conducted studies are also needed to assess these factors and the combination of different ages, ethnicity, and the effect of different laparoscopic nephroureterectomy procedures between the two groups, because this meta-analysis study could not answer whether they are related to the outcomes.

RETRACTED

In summary, the data recommend that laparoscopic nephroureterectomy in subjects with upper urinary tract urothelial carcinoma may decrease the risk of hospital stay, blood loss, transfusion need, and overall complication and prolong the operation time compared with open nephroureterectomy in subjects with upper urinary tract urothelial carcinoma. Further studies are needed to validate these findings.

### Limitations

There may be selection bias in this study because many studies found were omitted from the meta-analysis. The studies omitted did not fulfill the inclusion criteria of this meta-analysis. Also, we could not respond whether the outcomes are related to age, ethnicity, and the effect of different laparoscopic nephroureterectomy procedures between the two groups or not. The study designed to evaluate the association between the efficacy and safety of open nephroureterectomy compared with laparoscopic nephroureterectomy in the treatment of upper urinary tract urothelial carcinoma was based on data from previous studies, which might cause bias induced by incomplete details. The meta-analysis was based on 36 studies; 9 studies were small, ≤ 100. Variables including age, ethnicity, and nutritional status of subjects were also the possible bias-inducing factors. Some unpublished articles and missing data may cause a bias in the pooled effect. Also, the criteria of surgical treatment choice were not fully explained. Subjects were using different treatment schedules, the dosage of the anesthesia, sedation use, and health care systems. Also, the varying definition of recurrence-free survival, cancer-specific survival, and overall survival might cause biases. In addition, the pathological variables, the length of follow-up, the operation procedures, and the experience of the surgeons were not the same in the selected studies.

RETRACTED

## Conclusion

Laparoscopic nephroureterectomy in subjects with upper urinary tract urothelial carcinoma may have a longer operation time, shorter hospital stay, and lower blood loss, transfusion need, and overall complication compared with open nephroureterectomy, however, no significant difference was found between laparoscopic nephroureterectomy and open nephroureterectomy in subjects with upper urinary tract urothelial carcinoma in 2–5 years recurrence-free survival, 2–5 years cancer-specific survival, and 2–5 years overall survival. Though the analysis of the results should be done with caution due to the lower number of subjects in some of the studies evaluating each parameter in this meta-analysis, suggesting more studies relating the type of operation method, and postoperative results in subjects with upper urinary tract urothelial carcinoma to validate these findings.

## Data Availability Statement

The original contributions presented in the study are included in the article/supplementary material, further inquiries can be directed to the corresponding author/s.

## Author Contributions

BL: conception and design. GL, ZY, GC, YL, and BL: administrative support, provision of study materials or subjects, data analysis and interpretation, manuscript writing, and final approval of manuscript. GL, ZY, GC, and YL: collection and assembly of data. All authors contributed to the article and approved the submitted version.

## Conflict of Interest

The authors declare that the research was conducted in the absence of any commercial or financial relationships that could be construed as a potential conflict of interest.

## Publisher's Note

All claims expressed in this article are solely those of the authors and do not necessarily represent those of their affiliated organizations, or those of the publisher, the editors and the reviewers. Any product that may be evaluated in this article, or claim that may be made by its manufacturer, is not guaranteed or endorsed by the publisher.
